# The Favorable Effect of Mesenchymal Stem Cell Treatment on the Antioxidant Protective Mechanism in the Corneal Epithelium and Renewal of Corneal Optical Properties Changed after Alkali Burns

This article has been retracted.

**DOI:** 10.1155/2016/5843809

**Published:** 2016-01-05

**Authors:** Cestmir Cejka, Vladimir Holan, Peter Trosan, Alena Zajicova, Eliska Javorkova, Jitka Cejkova

**Affiliations:** ^1^Laboratory of Eye Histochemistry and Pharmacology, Institute of Experimental Medicine, Academy of Sciences of the Czech Republic, Videnska 1083, 14220 Prague 4, Czech Republic; ^2^Department of Transplantation Immunology, Institute of Experimental Medicine, Academy of Sciences of the Czech Republic, Videnska 1083, 14220 Prague 4, Czech Republic; ^3^Faculty of Natural Science, Charles University, Vinicna 7, 12843 Prague 2, Czech Republic

## Abstract

The aim of this study was to examine whether mesenchymal stem cells (MSCs) and/or corneal limbal epithelial stem cells (LSCs) influence restoration of an antioxidant protective mechanism in the corneal epithelium and renewal of corneal optical properties changed after alkali burns. The injured rabbit corneas (with 0.25 N NaOH) were untreated or treated with nanofiber scaffolds free of stem cells, with nanofiber scaffolds seeded with bone marrow MSCs (BM-MSCs), with adipose tissue MSCs (Ad-MSCs), or with LSCs. On day 15 following the injury, after BM-MSCs or LSCs nanofiber treatment (less after Ad-MSCs treatment) the expression of antioxidant enzymes was restored in the regenerated corneal epithelium and the expressions of matrix metalloproteinase 9 (MMP9), inducible nitric oxide synthase (iNOS), *α*-smooth muscle actin (*α*-SMA), transforming growth factor-*β*1 (TGF-*β*1), and vascular endothelial factor (VEGF) were low. The central corneal thickness (taken as an index of corneal hydration) increased after the injury and returned to levels before the injury. In injured untreated corneas the epithelium was absent and numerous cells revealed the expressions of iNOS, MMP9, *α*-SMA, TGF-*β*1, and VEGF. In conclusion, stem cell treatment accelerated regeneration of the corneal epithelium, restored the antioxidant protective mechanism, and renewed corneal optical properties.

## 1. Introduction

Alkali injury of the cornea threatens vision. Immediately after the alkali injury oxidative stress appears in the cornea, which precedes the corneal inflammatory response [1, 2]. Following alkali injury of the cornea or after irradiation of the cornea with UVB rays, the antioxidant/prooxidant imbalance appeared in the damaged corneal epithelium. The expression and activities of corneal antioxidant enzymes decreased, whereas the expression and activities of prooxidant enzymes remained at physiological levels or even increased [3, 4]. Reactive oxygen species (ROS) were insufficiently cleaved. According to Finkel and Holbrook [5] ROS can activate the transcription factor NF-kB, which then translocate to the nucleus to induce the production of proinflammatory cytokines, highly involved in the development of inflammation. ROS contribute to the induction of various enzymes, such as metalloproteinases, serine proteases, and nitric oxide synthases [6, 7]. Toxic oxygen and nitrogen products with proteolytic enzymes degrade the cornea [8, 9]. The immediate start of topical treatment of the alkali-injured eye with antioxidant H2-enriched irrigation solution and N-acetyl-L-cysteine [1] or with bone marrow mesenchymal stem cells (BM-MSCs) revealing antioxidant properties significantly suppressed intracorneal inflammation and corneal neovascularization [2]. It is well known that MSCs possess antioxidant properties [2, 10–13]. The beneficial antioxidant effects of MSCs may be explained by the findings that MSCs secrete superoxide dismutase [14]. Superoxide dismutase belongs to antioxidant enzymes that dismute toxic free radicals produced during inflammation [15].

To our knowledge, this is the first paper investigating the effects of bone marrow MSCs (BM-MSCs), adipose tissue MSCs (Ad-MSCs), or corneal limbal epithelial stem cells (LSCs) on the antioxidant protective mechanism in the regenerated corneal epithelium and on corneal optical properties evaluated by central corneal thickness (taken as an index of corneal hydration) and corneal transparency. We found that in contrast to the effect of nanofibers alone (MSCs-free), where profound enzymatic antioxidant/prooxidant imbalance was found in the corneal epithelium, after the treatment of injured corneas with BM-MSCs nanofibers or LSCs nanofibers (less after Ad-MSCs nanofibers), the enzymatic antioxidant protective mechanism was restored in the regenerated corneal epithelium. This was accompanied by the renewal of corneal optical properties and accelerated corneal healing.

## 2. Material and Methods

### 2.1. Preparation of Stem Cells

LSCs were obtained by enzyme digestion of rabbit limbal tissue as we have described in a mouse model [16]. In brief, limbal tissue was cut with scissors and subjected to 10 short (10 min each) trypsinization cycles. The released cells were harvested after each cycle, centrifuged (8 minutes at 250 g), and resuspended in RPMI 1640 medium (Sigma, St. Louis, MO) containing 10% fetal calf serum (FCS, Sigma), antibiotics (100 U/mL of penicillin, 100 *μ*g/mL of streptomycin), and 10 mM HEPES buffer. The cells were seeded in 25 cm^2^ tissue culture flasks (Corning, Schiphol-Rijk, Netherlands). For characterization of cells and for their transfer to the nanofiber scaffold, the cells growing in vitro for 2-3 weeks (3rd passage) were used.

BM-MSCs were isolated from femurs of rabbits. The bone marrow was flushed out, a single cell suspension was prepared by homogenization, and the cells were seeded at a concentration of 4 × 10^6^ cells/mL in Dulbecco's modified Eagle's medium (DMEM, Sigma) containing 10% FCS, antibiotics (100 U/mL of penicillin, 100 mg/mL of streptomycin), and 10 mM HEPES in 25 cm^2^ tissue culture flasks (Corning). After a 48-hour incubation, the nonadherent cells were washed out and the adherent cells were cultured with a regular exchange of the medium and passaging of the cells to maintain their optimal concentration. The cells were characterized and used after the 3rd passage.

Ad-MSCs were isolated from subcutaneous adipose tissue. The tissue was cut into small pieces with scissors and incubated in 1 mL of Hank's balanced salt solution containing 10 mg/mL of collagenase type I (Sigma) for 60 minutes at 37°C with gentle agitation. Then the collagenase was diluted with complete DMEM. The cells were filtered and centrifuged at 250 g for 8 minutes. The upper adipose layer was removed, and cells were centrifuged, resuspended in 6 mL of complete DMEM (4 × 10^6^ cells/mL), and seeded in 25 cm^2^ tissue culture flasks (Corning). After incubation for 48 hours, the cells were washed with a medium to remove nonadherent cells and cell debris and cultured under standard conditions. Ad-MSCs were used in passages 3-4.

### 2.2. Stem Cell Differentiation and Gene Expression

The ability of stem cells to differentiate into other cell types was determined according to the ability to differentiate into adipocytes using specific adipogenic medium containing 0.1 *μ*M dexamethasone, 0.5 mM 3-isobutyl-1-methylxanthine, 0.1 mM indomethacin, and 0.5 *μ*g/mL of insulin, as we described previously [17]. Differentiation of cells was confirmed by staining with Oil Red O.

The expression of genes for the immunoregulatory molecules indoleamine-2,3-dioxygenase (IDO), cyclooxygenase-2 (Cox-2), and transforming growth factor-*β* (TGF-*β*) was determined in unstimulated and lipopolysaccharide- (LPS-) stimulated MSCs and LSCs. In these experiments, the cells (4 × 10^4^ cells/well) were cultured in 700 *μ*L of DMEM for 48 hours in 24-well tissue culture plates (Corning) with or without 5 *μ*g/mL of LPS, and the expression of the genes was determined by real-time PCR, as we have described elsewhere [18].

### 2.3. Nanofiber Scaffold Preparation

The PLA polymer was purchased from Nature Works LLC (Minnetonka, Minneapolis, Minnesota, USA). This material was dissolved in chloroform at 7 weight percent (wt%), and two other solvents, 1,2-dichloroethane (29 wt%) and ethyl acetate (10 wt%) (both purchased from PENTA, Prague, Czech Republic), were added to this solution. The mixture was stirred until a homogenous polymer solution was obtained. The modified needleless Nanospider technology, in which polymeric jets are spontaneously formed from liquid surfaces on a rotating spinning electrode, was used to prepare the nanofibers. Nanofiber scaffolds were cut into squares (approximately 1.5 × 1.5 cm) and fixed into CellCrown24 inserts (Scaffdex). The inserts with nanofibers were transferred into 24-well tissue culture plates (Corning). Three × 10^5^ stem cells in a volume of 700 *μ*L of complete DMEM were transferred into each well. The plates were incubated for 24 hours to allow cells to adhere to the scaffold [19].

### 2.4. Alkali Injury of the Cornea in Experimental Animals and Nano Scaffold Transfer

Adult female New Zealand white rabbits (2.5–3.0 kg) were used in our experiments. The investigation was conducted according to the ARVO Statement on the Use of Animals in Ophthalmic and Vision Research. Rabbits were anesthetized by an intramuscular injection of Rometar (xylazinum hydrochloricum, Spofa, Prague, CR, 2%, 0.2 mL/kg body weight) and Narkamon (ketaminum hydrochloricum, Spofa, 5%, 1 mL/kg body weight).

Sodium hydroxide (0.25 N NaOH) was applied by means of dropping on the corneal surface (10 drops during 1 min); then the eyes were immediately rinsed with tap water. The animals were divided into five groups (each group contained six rabbits). In the first group of animals, the injured eyes were left without further treatment. In the second group drug-free nanofiber scaffolds were transferred onto the injured eyes and sutured to the conjunctiva and the eyelids closed. In the third group BM-MSCs nanofibers were transferred onto the injured corneal surface and sutured to the conjunctiva and the eyelids closed. In the fourth group Ad-MSCs nanofibers were transferred with cell side facing down on the alkali-injured corneal surface and sutured to the conjunctiva and the eyelids closed. In the fifth group LSCs nanofibers were transferred to the corneal surface and sutured to the conjunctiva and the eyelids closed.

The scaffolds were transferred onto the ocular surface immediately after the injury and sutured to the conjunctiva with four interrupted sutures using 11.0 Ethilon (Ethicon, Johnson & Johnson, Livingston, England). The eyelids were closed by tarsorrhaphy using 1 suture of Resolon 7.0 (Resorba, Nuremberg, Germany) for 72 hours. An ophthalmic ointment compound containing bacitracin and neomycin (Ophthalmo-Framykoin, Zentiva, Prague, Czech Republic) was applied. The nanofiber scaffolds were removed from the ocular surface on day 4 after the operation. After the alkali injury and awakening from the anesthesia, the rabbits were treated with analgesia (ketoprofen, 1.0 mg/kg i.m.) two times daily for five days. The animals were sacrificed following an i.v. injection of thiopental anesthesia (Thiopental, Spofa, 30 mg/kg) after premedication with an intramuscular injection of Rometar/Narkamon on day 15 after the injury. In all experiments with alkali injury, the corneas of healthy rabbit eyes served as controls. Photographs of the corneas were taken throughout the whole experiment.

### 2.5. Microscopical Examinations

After sacrificing the animals, the eyes were enucleated and the anterior eye segments dissected out and quenched in light petroleum chilled with an acetone-dry ice mixture. Sections were cut on a cryostat and transferred to glass slides. Subsequently, the cryostat sections were fixed in acetone at 4°C for 5 minutes. For the immunohistochemical localization of xanthine oxidase (XOX), superoxide dismutase (SOD), glutathione peroxidase (GPX), catalase (CAT), *α*-smooth muscle actin (*α*-SMA), inducible nitric oxide synthase (iNOS), matrix metalloproteinase-9 (MMP9), interleukin-6 (IL-6), and vascular endothelial growth factor (VEGF), the following primary antibodies were used: mouse monoclonal anti-xanthine oxidase Ab-2 (NeoMarkers, Fremont, CA, USA), mouse monoclonal anti-superoxide dismutase, sheep polyclonal anti-catalase, sheep polyclonal anti-glutathione peroxidase (Biogenesis, Poole, UK), goat polyclonal anti-matrix metalloproteinase-9 (Santa Cruz Biotechnology, Santa Cruz, CA, USA), mouse monoclonal anti-*α*-SMA (Sigma, Saint Louis, MO, USA), mouse monoclonal anti-human iNOS (Biosciences, San Jose, CA, USA), goat polyclonal anti-MMP9 (Santa Cruz Biotechnology, Santa Cruz, CA, USA), mouse monoclonal anti-IL-6 (Abcam, Cambridge, UK), and mouse monoclonal anti-VEGF (Abcam, Cambridge, UK). The binding of the primary antibodies was demonstrated using the HRP/DAB Ultra Vision detection system (Thermo Scientific, Fremont, CA) following the instructions of the manufacturer: hydrogen peroxide block (15 minutes), ultra V block (5 minutes), primary antibody incubation (60 minutes), biotinylated goat anti-mouse IgG (Lab Vision, Fremont, CA) or donkey anti-goat IgG (Santa Cruz Biotechnology) secondary antibody incubation (10 min), and peroxidase-labeled streptavidin incubation (10 minutes). Visualization was performed using a freshly prepared DAB substrate-chromogen solution. Cryostat sections in which the primary antibodies were omitted from the incubation media served as negative controls. Some sections were counterstained with Mayer's hematoxylin.

### 2.6. Determination of Corneal Thickness

Changes of corneal optical properties after the injury and during healing were evaluated by measuring the central corneal thickness (taken as an index of corneal hydration) [20]. The central corneal thickness was measured in anesthetized animals using an ultrasonic pachymeter SP-100 (Tomey Corporation, Nagoya, Japan) in the corneal center. The corneal thickness was measured in the same corneas before alkali injury (corneas of healthy eyes) and five and fifteen days after the injury (all experimental groups). Each cornea was measured four times and the mean value of the thickness (in *μ*m) was computed.

### 2.7. Evaluation of Corneal Neovascularization and Transparency

For evaluation of corneal neovascularization, the number of vessels was counted in each of 60° sectors of the corneal surface. The mean value and standard deviation were counted from five measurements. This procedure was applied for every eye from a matching group of eyes (control, injured untreated, injured and treated with drug-free nanofibers, and injured and treated with MSCs nanofibers or with Ad-MSCs nanofibers or with LSCs nanofibers).

### 2.8. Detection of Gene Expression by Real-Time PCR

The expression of genes for TGF-*β*1, VEGF, and iNOS in control and treated corneas was determined by quantitative real-time polymerase chain reaction (PCR). Corneas were excised using Vannas scissors, transferred into Eppendorf tubes, and immediately frozen. The frozen corneal tissue was then homogenized and added in 500 *μ*L of TRI Reagent (Molecular Research Center, Cincinnati, OH) for the RNA isolation. The details of RNA isolation, transcription, and the PCR parameters have been described previously [21]. In brief, total RNA was extracted using TRI Reagent according to the manufacturer's instructions. One *μ*g of total RNA was treated using deoxyribonuclease I (Promega) and subsequently used for reverse transcription. The first-strand cDNA was synthesized using random primers (Promega, Madison, WI) in a total reaction volume of 25 *μ*L, using M-MLV Reverse Transcriptase (Promega).

Quantitative real-time PCR was performed in a StepOnePlus real-time PCR system (Applied Biosystems). The relative quantification model with efficiency correction was applied to calculate the expression of the target gene in comparison with GAPDH used as the housekeeping gene. The following primers were used for amplification: GAPDH: 5′-CCCAACGTGTCTGTCGTG (sense), 5′-CCGACCCAGACGTACAGC (antisense), iNOS: 5′-AGGGAGTGTTGTTCCAGGTG (sense), 5′-TCCTCAACCTGCTCCTCACT (antisense), TGF-*β*1: 5′-GCCTGCAAGTGCTCAAGTTAC (sense), 5′-TGCTGCATTTCTGGTACAGC (antisense), and VEGF: 5′-CGAGACCTTGGTGGACATCT (sense), 5′-ATCTGCATGGTGACGTTGAA (antisense). The PCR parameters included denaturation at 95°C for 3 min, then 40 cycles at 95°C for 20 s, annealing at 60°C for 30 s, and elongation at 72°C for 30 s. Fluorescence data were collected at each cycle after an elongation step at 80°C for 5 s and were analyzed on the StepOne Software, version 2.2.2 (Applied Biosystems). Each individual experiment was done in triplicate.

### 2.9. Statistics

An analysis of the data showed normal distribution and the results are expressed as mean ± SD. Comparisons between the two groups were made by Student's* t*-test, and multiple comparisons were analyzed by ANOVA. A value of *P* < 0.05 was considered statistically significant.

## 3. Results

### 3.1. Differentiation and Gene Expression of Rabbit MSCs and LSCs

When all three cell types were cultured in a specific adipogenic differentiation medium, the highest differentiation potential was recorded in BM-MSCs, as demonstrated microscopically (Figure 1(a)). To test the ability of BM-MSCs, Ad-MSCs, and LSCs to express genes for the basic immunoregulatory molecules, the cells were cultured for 48 hours unstimulated or stimulated with LPS and the expression of genes for IDO-2, iNOS, and Cox-2 was determined by real-time PCR. As demonstrated in Figure 1(b), the gene for TGF-*β*1 was expressed spontaneously and comparably in all cell types, while the genes for IDO and Cox-2 were expressed preferentially in only some cell populations or only after stimulation with LPS.

### 3.2. Immunohistochemical Detection of SOD, XOX, MMP9, and iNOS and Gene Expression of iNOS in the Alkali-Injured and Stem Cell Treated Corneas (Day 15 after the Injury)

The expressions of SOD and XOX were balanced in injured corneas treated with BM-MSCs nanofibers (Figures 2(c) and 2(d)) and LSCs nanofibers (Figures 2(g) and 2(h)), similar to the control (healthy corneas) (Figures 2(i) and 2(j)). In injured corneas treated with Ad-MSCs, the expression of SOD (Figure 2(e)) was decreased compared to controls (Figure 2(i)). The expression of SOD was also decreased (compared to controls) in injured corneas treated with cell-free nanofibers (Figure 2(a)). Similar results (as with SOD) were obtained with the expression of CAT and GPX (images not shown). Also in these cases the balance between the expressions of CAT and XOX and GPX and XOX was obtained only in injured corneas treated with BM-MSCs nanofibers or LSCs nanofibers. The expressions of CAT and GPX were decreased (compared to controls) after the treatment of injured corneas with Ad-MSCs or Nano free of MSCs. The expression of MMP9 (Figure 3(a)) or iNOS (Figure 3(b)) was high in injured untreated corneas and only less decreased in injured corneas treated with cell-free nanofibers (Figures 3(c) and 3(d)). However, the treatment of injured corneas with BM-MSCs nanofibers (Figures 3(e) and 3(f)) or with LSCs nanofibers (Figures 3(i) and 3(j)) (less after Ad-MSCs nanofibers, Figures 3(g) and 3(h)) suppressed the expression of MMP9 and iNOS in corneas. The expression of MMP9 (Figure 3(k)) was very low in control corneas and the expression of iNOS (Figure 3(l)) was absent. The expression of genes for iNOS in healthy, injured untreated, and injured treated corneas was quantified by real-time PCR (Figure 3(m)). In accordance with the results from immunohistochemistry, treatment of injured corneas with BM-MSC nanofibers or LSC-seeded nanofiber scaffolds decreased the iNOS expressions.

### 3.3. Immunohistochemical Detection of *α*-SMA and VEGF and Gene Expression of TGF-*β* in Alkali-Injured and Stem Cell Treated Corneas (Day 15 after the Injury)

In injured untreated corneas (Figure 4(a)) and corneas treated with stem-cell-free nanofibers (Figure 4(b)) the expression of *α*-SMA was high, whereas, in injured corneas treated with BM-MSCs nanofibers (Figure 4(c)), with LSCs (Figure 4(e)), or with Ad-MSCs nanofibers (Figure 4(d)), the expressions were low. In control (healthy) corneas (Figure 4(f)) the expression of *α*-SMA was absent. The expression of genes for TGF-*β*1 in healthy and injured untreated and treated corneas with stem cells was quantified by real-time PCR (Figure 4(g)). The treatment of injured corneas with stem cells decreased the expression of TGF-*β*1. The expression of VEGF was very low in healthy control corneas (Figure 5(f)). On day 15 after the injury, the expression of VEGF was high in untreated corneas (Figure 5(a)) and was only less decreased in corneas treated with cell-free nanofiber scaffold (Figure 5(b)). The treatment of injured corneas with Ad-MSC-seeded nanofibers reduced VEGF expression (Figure 5(d)). The highest reduction of VEGF expression was seen in corneas treated with BM-MSCs nanofiber scaffolds (Figure 5(c)) or LSCs nanofibers (Figure 5(e)). The expression of genes for VEGF in control (healthy), injured untreated, and injured treated corneas was quantified by real-time PCR (Figure 5(g)). The treatment of injured corneas with stem-cell-seeded nanofiber scaffolds significantly decreased the expression of VEGF.

### 3.4. Corneal Opacity of Alkali-Injured and Stem Cell Treated Eyes

Representative photographs of healthy, injured, and treated eyes are shown in Figure 6. In comparison with the healthy control eyes (Figure 6(a)), corneas of injured eyes became opalescent following the injury (Figure 6(b)) and remained opalescent and highly vascularized on day 15 after the injury (Figure 6(d)). The eye covered with nanofiber scaffold immediately after the injury is shown in Figure 6(c). Some improvement of corneas was observed on day 15 after the injury in eyes treated with cell-free nanofiber scaffold (Figure 6(e)); however, corneas were vascularized. In the eyes treated with stem-cell-seeded nanofibers, the corneal opacity was decreased and corneal neovascularization was apparently less expressed (Figures 6(f)–6(h)) with the best therapeutic effects of the treatment with BM-MSCs (Figure 6(f)) or with LSCs (Figure 6(h)). Quantification of corneal neovascularization is summarized in Figure 6(i). The number of vessels was high in injured untreated corneas and was partially reduced in injured corneas treated with cell-free nanofibers. Treatment of injured corneas with nanofiber scaffolds seeded with all three types of stem cells significantly decreased corneal neovascularization. The highest decrease was found in injured corneas treated with nanofiber scaffolds seeded with BM-MSCs or with LSCs.

### 3.5. Central Corneal Thickness after Alkali Injury and Treatment with Stem Cells (Figure 7)

Shortly after alkali injury, the central corneal thickness increased more than twice (compared to levels before injury, day 0) and remained high on day 5 in untreated corneas or in corneas treated with cell-free nanofiber scaffold. The central corneal thickness was significantly reduced already on day 5 in corneas treated with nanofiber scaffolds seeded with stem cells. On day 15 after injury, the corneal thickness remained increased in untreated injured corneas but was profoundly decreased in corneas treated with stem-cell-seeded nanofibers. On day 15 after the injury, in corneas treated with nanofiber scaffolds seeded with BM-MSCs or LSCs, the corneal thickness returned to the values before injury (day 0).

## 4. Discussion

In this paper, the stem cells were incubated and transferred onto the damaged corneal surface with CsA-loaded nanofiber scaffolds. The nanofiber scaffolds are biocompatible and have good mechanical properties to fixate on the ocular surface. The stem cells migrate from the scaffolds onto the ocular surface and support corneal healing [22]. Moreover, CsA-loaded nanofibers are synthetic and for this reason more suitable in many cases than biomaterials, such as collagen sheets or amniotic membrane. These biomaterials have some limitations, such as enzymatic digestion of collagen sheets [23] or the presence of anti- as well as proinflammatory cytokines (IL-6, IL-8) or metalloproteinases in amniotic membranes which may in some cases controversially contribute to corneal melting [24]. Using CsA-loaded nanofibers, our results show that the treatment of alkali-injured corneas with BM-MSCs nanofibers or LSCs nanofibers (less with Ad-MSCs nanofibers) accelerated corneal reepithelialization and restored the antioxidant/prooxidant balance in the regenerated corneal epithelium. This was accompanied by corneal healing with renewed optical properties and highly reduced neovascularization.

The antioxidant mechanism located in the corneal epithelium is very important for the protection of the cornea against toxic environmental influences. After the injury with alkali or irradiation of the cornea with UVB rays, the levels of corneal antioxidant enzymes (SOD, CAT, and GPX) decreased in the corneal epithelium, whereas the levels of prooxidant enzymes, oxidases that generate ROS, with the most important role of XOX, remained at physiological levels or even increased [2–4]. ROS generated in high numbers were insufficiently cleaved. This was dangerous to the cornea because ROS induce proinflammatory cytokine generation leading to the increased expression and activation of destructive enzymes damaging the cornea [25]. According to the concentration of alkali and extent of injury, corneas ulcerate or perforate during 2 to 3 weeks after the injury or corneas slowly heal with untransparent scar formation [26]. From our previous studies (unpublished results) it followed that, after the injury of rabbit corneas with 0.25 N NaOH (by means of dropping on the corneal surface), the corneal epithelium was lost after the injury and during the subsequent 15 days the epithelium was not regenerated in untreated injured corneas. Therefore, this time interval was chosen in this study (as the end of experiment) using a similar concentration of alkali and mode of application. We found that on day 15 the after the injury the untreated corneas were not reepithelialized. This was in contrast to injured corneas treated with nanofibers alone (MSCs-free) which were reepithelialized; however, the expressions of antioxidant enzymes were decreased in the regenerated corneal epithelium (compared to healthy control corneas). In contrast, after BM-MSCs nanofiber or LSCs nanofiber treatment the expressions of antioxidant enzymes were restored and balanced with prooxidant enzymes in the epithelium, similar to the control (healthy) corneas (Figure 2).

In this study, BM-MSCs, Ad-MSCs, and LSCs were prepared from the same rabbit and their growth, differentiation properties, and the ability to produce immunoregulatory and growth factors were compared (Figure 1). Besides the immunomodulatory and anti-inflammatory properties of MSCs, these stem cells reveal important antioxidant effects. MSCs can exert direct antioxidant activities through the secretion of antioxidant molecules. They secrete the extracellular antioxidant molecule superoxide dismutase 3 (SOD3) [14, 27]. The superoxide dismutase family member SOD3 is the only antioxidant enzyme that scavenges superoxide in the extracellular space and reduces the formation of toxic oxygen and nitrogen products, such as the hydroxyl radical and peroxynitrite. In our experiments stem cells on nanofiber scaffolds were transferred immediately after the injury to the damaged ocular surface. It is suggested that the SOD3 of stem cells cleaved ROS generated, for example, by XOX because both SOD3 and ROS were released extracellularly [4]. This may be one mechanism decreasing the amount of ROS and supporting corneal reepithelialization and healing. In injured corneas treated with stem cells seeded on nanofiber scaffolds, the expression and levels of MMP9, iNOS, *α*-SMA, TGF-*β*1, and VEGF were significantly decreased compared to untreated injured corneas or injured corneas treated with Nano free of MSCs (Figures 3–5). It has been demonstrated in a variety of experimental studies that SOD3 can attenuate tissue damage and inflammation [28, 29]. The ability of transplanted LSCs to regenerate corneal epithelium [30] is well known. This is also shown in our study. However, we first demonstrate in this study the renewal of the expression of antioxidant enzymes in the regenerated corneal epithelium after the treatment of alkali-injured corneas with stem cells.

## 5. Conclusions

BM-MSCs nanofibers and LSCs nanofibers (less Ad-MSCs nanofibers), transferred onto the damaged corneal surface immediately after the injury, accelerated corneal reepithelialization and restored the antioxidant/prooxidant balance in the regenerated corneal epithelium. Corneal inflammation was suppressed and corneal neovascularization reduced. The central corneal thickness (taken as an index of corneal hydration) reached levels before injury. Corneal optical properties were renewed to a large extent. Although there are some differences between the human and rabbit cornea in the recovering of endothelial function (faster in rabbits thanks to cell proliferation), the efficacy of stem cell treatment of alkali-injured cornea on the renewal of physiological levels of corneal hydration and on the restoration of transparency compared to untreated injured corneas or injured corneas treated with nanofibers free of cells was clearly shown in our rabbit model.

## Figures and Tables

**Figure 1:** The ability of cells to differentiate into adipocytes was characterized microscopically ((a) upper: undifferentiated cells; lower: cells in differentiation medium). Expression of genes for immunoregulatory molecules by BM-MSCs, Ad-MSCs, and LSCs (b). The cells were cultured for 48 hours unstimulated or stimulated with LPS and the expression of genes for IDO, TGF-*β*, and Cox-2 was determined by real-time PCR. Each bar represents the mean ± SD from 5 determinations.

**Figure 2:** The immunohistochemical detection of SOD and XOX in the corneal epithelium in injured and stem cell treated corneas on day 15 after the injury. In BM-MSCs treated corneas (c, d) and LSCs treated corneas (g, h), expressions of SOD and XOX are relatively high and balanced, similar to the control corneas (i, j). In contrast, in Ad-MSCs treated corneas (e, f) and Nano-treated corneas (a, b) the expressions of SOD are decreased compared to controls (i). Scale bars: 50 *μ*m.

**Figure 3:** The expression of MMP9 and iNOS in injured and stem cell treated corneas on day 15 after the injury. The expression of MMP9 (a) and iNOS (b) in untreated corneas without epithelium and in Nano-treated reepithelialized corneas (c, d) is high and decreases in Ad-MSCs treated corneas (g, h). In corneas treated with BM-MSCs (e, f) or LSCs (i, j) the expressions of MMP9 are low and the expression of iNOS is nearly absent, similar to the control cornea (k, l). The corneal sections are counterstained with hematoxylin. Scale bars: 50 *μ*m. The expression of genes for iNOS (m) on day 15 after the injury was determined by real-time PCR. Each bar represents the mean ± SD from 6 individual corneas. The values with asterisks represent statistically significant (^*∗*^ *P* < 0.05) difference from untreated injured corneas.

**Figure 4:** The expression of *α*-SMA and TGF-*β*1 in injured and stem cell treated corneas on day 15 after the injury. The expression of *α*-SMA is high in untreated (a) and Nano-treated (b) corneas, whereas in corneas treated with BM-MSCs (c), Ad-MSCs (d), and LSCs (e) it is low. Compare with control cornea (f), where the expression of *α*-SMA is absent. The corneal sections are counterstained with hematoxylin. Scale bars: 50 *μ*m. The expression of genes for TGF-*β*1 (g) on day 15 after the injury was determined by real-time PCR. Each bar represents the mean ± SD from 6 individual corneas. The values with asterisks represent a statistically significant (^*∗*^ *P* < 0.05, ^*∗∗*^ *P* < 0.01) difference from untreated injured corneas.

**Figure 5:** The expression of VEGF in injured and stem cell treated corneas on day 15 after the injury. VEGF expression is high in untreated corneas (a) and Nano-treated corneas (b) and less expressed in Ad-MSCs treated corneas (d). After the treatment of corneas with BM-MSCs (c) and LSCs (e), the expression of VEGF is low. In control corneas (f) the expression of VEGF is absent. The sections are counterstained with hematoxylin. Scale bars: 50 *μ*m. The expression of genes for VEGF (g) on day 15 after the injury was determined by real-time PCR. Each bar represents the mean ± SD from 6 individual corneas. The values with asterisks represent a statistically significant (^*∗*^ *P* < 0.05) difference from untreated injured corneas.

**Figure 6:** Corneal opacity of alkali-injured and stem cell treated eyes. Representative photographs show a control healthy eye (a), alkali-injured eye (immediately after the injury) (b), the injured eye with sutured nanofiber scaffold (immediately after the injury) (c), and injured eyes on day 15 after the injury which were untreated (d) or treated with cell-free nanofiber scaffold (e) or with nanofiber scaffolds seeded with BM-MSCs (f), Ad-MSCs (g), or LSCs (h). Corneal neovascularization is strongly expressed in untreated corneas ((d) arrows) and highly suppressed in corneas treated with nanofiber scaffolds BM-MSCs (f) and LSCs (h). The quantification of corneal neovascularization is shown in (i). Each bar represents the mean ± SD from 6 corneas. The values with asterisks are significantly different (^*∗∗∗*^ *P* < 0.001) from untreated injured corneas.

**Figure 7:** Central corneal thickness of healthy, alkali-injured, and stem cell treated corneas. The corneas were injured with alkali and untreated or treated with nanofiber scaffold alone (Nano) or with nanofiber scaffolds seeded with BM-MSCs, Ad-MSCs, or LSCs. Central corneal thickness was measured in the same rabbit before injury (day 0) and on days 5 and 15 after the injury. Each bar represents the mean ± SD from 6 corneas. The values (black asterisks) for day 5 are statistically different from untreated injured corneas on day 5; similarly, the values for day 15 (black asterisks) are statistically different from untreated injured corneas on day 15 (^*∗*^ *P* < 0.05, ^*∗∗∗*^ *P* < 0.001) (n.s.: not significant). The values for day 15 (red asterisks) are statistically different from the values before injury, day 0 (^*∗∗∗*^ *P* < 0.001) (n.s.: not significant).

## Abbreviations

BM-MSCs: Bone marrow mesenchymal stem cells
Ad-MSCs: Adipose tissue mesenchymal stem cells
LSCs: Limbal corneal epithelial stem cells
ROS: Reactive oxygen species
iNOS: Inducible nitric oxide synthase
MMP9: Matrix metalloproteinase-9
*α*-SMA: Alpha-smooth muscle actin
TGF-*β*1: Transforming growth factor-beta 1
VEGF: Vascular endothelial growth factor.
